The article "Chronic Recurrent Multifocal Osteomyelitis with Concomitant Features of Juvenile Idiopathic Arthritis" was retracted in 2014. Reason: missing or withdrawn patient consent.

# Chronic Recurrent Multifocal Osteomyelitis with Concomitant Features of Juvenile Idiopathic Arthritis

**DOI:** 10.1155/2011/210795

**Published:** 2011-12-29

**Authors:** Elena Tsitsami, Vasiliki Dermentzoglou, Mary Moschovi, George P. Chrousos

**Affiliations:** ^1^Pediatric Rheumatology Unit, 1st Department of Pediatrics, Children's Hospital Aghia Sophia, University of Athens, 115 27 Athens, Greece; ^2^Department of Radiology, Children's Hospital Aghia Sophia, 115 27 Athens, Greece; ^3^Hematology Oncology Unit, 1st Department of Pediatrics, Children's Hospital Aghia Sophia, University of Athens, 115 27 Athens, Greece; ^4^1st Department of Pediatrics, Children's Hospital Aghia Sophia, University of Athens, 115 27 Athens, Greece

## Abstract

We report a case of a 13-year-old girl with chronic recurrent multifocal osteomyelitis (CRMO) who developed severe arthritis in four different joints within the first year from the onset of the disease. Her multiple vertebrae lesions showed significant amelioration after a 2-month treatment with prednisolone. In parallel, the initial severe symmetrical arthritis of both knees showing overt synovitis and joint effusion, in the absence of lesions in the metaphyses of the femur or the tibia, responded remarkably well in intra-articular triamcinolone hexacetonide injections. However, upon discontinuation of prednisolone, the patient developed severe arthritis of her right ankle and the proximal interphalangeal joint of her right middle finger. Thus, prednisolone was reinitiated combined with methotrexate, and the patient went into remission, which persists one year after prednisolone tapering. The appearance of arthritis in both knees in the absence of bone lesions and the emergence of severe arthritis of the ankle after remission of spinal bone lesions suggest that CRMO and juvenile idiopathic arthritis may coexist and be causally related.

## 1. Introduction

Chronic recurrent multifocal osteomyelitis (CRMO) or CRMO syndrome (OMIM no. 259680) is a rare inflammatory bone disease presenting usually early in life (*∼*10 years of age) although adults with CRMO have been described. It shares many features with and is, therefore, regarded to be the pediatric subset of SAPHO (synovitis, acne, pustulosis, hyperostosis, and osteitis) syndrome considered together to constitute the unique disease spectrum of chronic nonbacterial osteomyelitis (CNO). Accordingly, CRMO syndrome is characterized by multiple foci of nonbacterial osteomyelitis appearing radiologically as a mixture of osteolytic/sclerotic lesions. It presents as bone pains with or without fever, has an unpredictable course alternating between exacerbations and spontaneous remission, and is frequently associated with other inflammatory and/or autoimmune conditions [1, 2].

The article "Chronic Recurrent Multifocal Osteomyelitis with Concomitant Features of Juvenile Idiopathic Arthritis" was retracted in 2014. Reason: missing or withdrawn patient consent.

The underlying defect and the pathogenesis of CRMO are largely unknown. Based on the finding that spontaneous recessive mutations in *Pstpip2 *(a murine gene encoding a protein homologous to the PAPA-pyogenic arthritis, pyoderma gangrenosum, and acne-syndrome protein PSTPIP1) cause, in the cmo mouse model, an autoinflammatory bone disease most closely resembling CRMO [3, 4], the later is considered as an autoinflammatory disorder [5]. Despite the fact that the human *PSTPIP2* gene is encoded within a genomic interval found to be associated with sporadic CRMO by transmission disequilibrium testing [6], no PSTPIP2 mutations have been as yet identified in CRMO syndrome.

As a result of its unknown etiology, diagnostic tests specific for CRMO do not exist, patients seem to be underdiagnosed, and its treatment is still empiric and not always successful. The histologic findings in bone biopsies are nonspecific, showing inflammatory changes with granulocytic infiltration. The situation is further confused due to the various classifications under which the syndrome appears in the literature. Beyond its already mentioned relation with SAPHO syndrome and based on the recurrent purulent manifestations involving joints, eye, skin, and bones, CRMO is classified amongst pyogenic autoinflammatory disorders, along with PAPA and Majeed syndromes [7]. On the other hand, several clinicians, looking at clinical, radiological, and histological findings, assume a common pathway for the different acute and chronic diseases associated with osteitis [8, 9]. In this context, the diagnostic criteria for nonbacterial osteomyelitis (acute and chronic) proposed by Jansson et al. [2], based on the analysis of a series of 89 patients with sterile bone inflammation (39 with CRMO without arthritis at first presentation), are expected to better discriminate CRMO patients among those with similar clinical and radiologic presentation.

This case report describes a 13-year-old girl with CRMO who, early after her initial presentation, developed polyarthritis that is incompatible with the as yet described physical history of the syndrome. This interesting fact brings not easily answerable questions about a possible coexistence of CRMO with juvenile idiopathic arthritis (JIA) as well as about an underlying autoinflammatory process able occasionally to give rise in a wider spectrum of symptoms, including polyarthritis.

## 2. Case Presentation

In June 2010, a previously healthy, 13-year-old girl initially presented to a local hospital with a three-month history of dorsal spine pain. At the time of presentation, physical examination revealed nothing remarkable, except arthritis of the left knee. No cutaneous involvement was noted. Laboratory test results, including bone marrow aspiration smear, were normal except for elevated ESR (33 mm/h) and CRP (9 mg/L), and a titer of antinuclear antibodies of 1 : 160. Despite magnetic resonance imaging (MRI) showing characteristic lesions (Figure 1), the diagnosis of CRMO was not considered, and the patient was hospitalized on several occasions for diagnostic investigation.

The article "Chronic Recurrent Multifocal Osteomyelitis with Concomitant Features of Juvenile Idiopathic Arthritis" was retracted in 2014. Reason: missing or withdrawn patient consent.

During the subsequent 6 months, the initial symptoms of the patient were worsening, and she therefore underwent an arthroscopy of the left knee and an open vertebral biopsy. Neither synovium nor vertebral biopsies provided any conclusive histopathologic features except a nonspecific chronic inflammatory process, while their standard cultures failed to identify any causal microorganism. All extensive investigation of infectious agents was negative. Based on a working diagnosis of bacterial osteomyelitis and septic arthritis, antibiotics, including amoxicillin/clavulanate potassium, ceftriaxone, and cefuroxime, were unsuccessfully administered, and the patient, in December 2010, was referred to our Pediatric Rheumatology Unit.

At that time, the patient was in bad general condition. She was febrile (39.5°C) and unable to remain standing for more than a few minutes. Physical examination showed severe muscular atrophy in both of the legs, slight dorsal scoliosis with convexity to the right and exacerbated arthritis of the left knee. The remainder of the examination was normal. There were no cutaneous lesions or lymphadenopathy and there was not family history of a chronic inflammatory disorder (psoriasis, inflammatory bowel disease, inflammatory arthritis severe acne, or any other).

Ultrasound examination and MRI demonstrated synovitis and joint effusion in both knees, most prominent in the left (Figure 2). MRI of the knees did not detect bone lesions in the distal femur or the proximal tibia (Figures 2(a), 2(c)). Bone scan showed increased uptake mainly in both knees, in thoracic vertebrae (T5, T6), in the left hip, and in the manubrium and body of the sternum (Figure 3). A new MRI of the spine showed again several vertebrae lesions of the cervical, thoracic, and lumbar spine with no evidence of deterioration or improvement. The lesions did not cross intervertebral discs as can occur in infection. The ESR was 68 mm/h, CRP was 134 mg/L, leukocytes were 7.410/*μ*L and anti-TPO antibodies were 90 IU/mL. HLA-B27 was absent.

Despite the inconclusive information provided by the previous histopathologic evaluation of the vertebral and synovial biopsies, as neither universal polymerase chain reaction to amplify eubacterial and mycobacterial genes, nor immunohistochemical examination were performed, further invasive diagnostic approach was avoided due to the bad general condition of the patient. Taking into account the failure of antibiotic treatments as well as the fact that the case was fulfilling the criteria of Jansson et al. [2], the diagnosis of CRMO was assumed. Treatment with indomethacin (2 mg/kg/day) was started, while intra-articular triamcinolone hexacetonide injections (40 mg) were performed in both knees. After 24 hours, the patient became afebrile and able to stand up and started walking. Concomitantly, however, she started complaining of headache that was attributed to indomethacin. Therefore, indomethacin was discontinued and prednisolone (1 mg/kg/day) was initiated. The patient responded remarkably well and, over the following weeks, she returned to her normal physical activity.

The article "Chronic Recurrent Multifocal Osteomyelitis with Concomitant Features of Juvenile Idiopathic Arthritis" was retracted in 2014. Reason: missing or withdrawn patient consent.

The prednisolone was gradually tapered and discontinued two months after the initiation. At that time, that is, one year after the appearance of the disease, the patient was reevaluated. She was in good general condition, the spinal MRI showed significant amelioration of bone lesions most of which had completely disappeared (Figure 4), and the US examination of both knees did not reveal findings of arthritis. However, she was complaining of pain and edema in the proximal phalanx of her right middle finger as well as in her right ankle. Therefore, prednisolone was reinitiated combined with methotrexate, and the patient went into remission, which persisted after prednisolone tapering and discontinuation.

## 3. Discussion

The diagnosis of CRMO is hampered by the lack of a specific diagnostic test and is essentially one of exclusions. Infective osteomyelitis, malignancy, and Langerhans' cell histiocytosis are the main differential diagnoses [10]. JIA cannot be excluded from the differential diagnosis [11], since in a recent report by Beck et al. [12], at the time of diagnosis, arthritis has been noted in as many as 38%, morning stiffness in 16.2%, functional impairment of legs in 43.2%, and asymmetry of extremities/thorax in 37.8% out of a series of 37 children patients. This high incidence of arthritis is not astonishing, bearing in mind that it affects always joints adjacent to the bone lesions as well as that metaphyses or metaphyseal equivalents are the most common sites of disease, accounting for approximately 75% of all lesions [13]. The arthritis of CRMO seems to be accompanied by mild synovitis and/or joint effusion although, to the best of our knowledge, exact data about their degree are lacking from the literature.

The article "Chronic Recurrent Multifocal Osteomyelitis with Concomitant Features of Juvenile Idiopathic Arthritis" was retracted in 2014. Reason: missing or withdrawn patient consent.

Due to the presence of the characteristic for CRMO multiple bone lesions, there was no difficulty to differentiate the case reported herein from JIA. However, the presence of severe symmetrical arthritis of the knees in the absence of lesions in the metaphyses of the femur or the tibia as well as the emergence of arthritis of the right ankle and the right proximal interphalangeal joint after the remission of spinal lesions is quite interesting. Furthermore, the severe muscular atrophy in both of the legs with which the patient presented implies that arthritis of the knees was initiated long before the appearance of CRMO lesions and was possibly not perceived or overridden by the dorsal spine pain. A suspicion of possible coincidence of the two diseases is therefore arisen, that necessitates a closer followup of the patient. Nevertheless, from the pathophysiological point of view and assuming an autoinflammatory nature of both disorders, this would be a simply rhetoric question, since a common autoinflammatory process could occasionally give rise in a brooder than the usual spectrum of CRMO symptoms, including polyarthritis.

It is also worth mentioning that, as in the case of our patient, improvement of CRMO arthritis by intra-articular corticosteroid injections has been also previously attempted [14]. Finally, the appearance of arthritis very early in the disease course of our patient deterred us from the major differential diagnosis of Langerhans' cell histiocytosis. Histiocytic oligoarthritis is a very rare finding of the later condition [15].

Even though JIA does not represent the major differential diagnosis of CRMO, the emergence of arthritis is not uncommon during the protracted course of the syndrome [16]. Moreover, evolution into enthesitis-related arthritis or spondyloarthropathy has been documented in children and young adults [16–18] underlining the need for long-term followup. However, the management of the reported patient before her referral to our unit indicates that a high index of suspicion is needed to diagnose CRMO syndrome, in order for misdiagnoses of infection and neoplasm, and unnecessary aggressive surgical and antibiotic therapy to be avoided.

## Figures and Tables

**Figure 1:** MRI of the spine at the disease presentation. Multiple vertebrae lesions are demonstrated in the cervical, thoracic, and lumbar spine, which exhibit increased signal intensity on sagittal T2-weighted images (a), (b), and (c). The appearance of the intervertebral discs is normal.

**Figure 2:** MRI and US of the left knee at the disease presentation. T2-weighted sagittal image (a) and US (b) demonstrated synovial thickening with increased vascularity (b) and joint effusion. The signal intensity of the distal femur and proximal tibia is normal (a), (c).

The article "Chronic Recurrent Multifocal Osteomyelitis with Concomitant Features of Juvenile Idiopathic Arthritis" was retracted in 2014. Reason: missing or withdrawn patient consent.

**Figure 3:** Bone scan at the disease presentation. Since the radiological investigation for bone lesions in this area proved negative, the increased uptake in both knees (a) was attributed to synovitis. Increased uptake was also demonstrated in the sternum (manubrium and body synchondrosis) (b), in thoracic vertebrae (c), and in the left hip (d).

**Figure 4:** MRI of the spine one year from the disease presentation.
